The article "Icariin Ameliorates Palmitate-Induced Insulin Resistance Through Reducing Thioredoxin-Interacting Protein (TXNIP) and Suppressing ER Stress in C2C12 Myotubes" was retracted in 2023. Reasons: duplicated images; unreliable data; unreliable results or conclusions; concerns about the images.

# Icariin Ameliorates Palmitate-Induced Insulin Resistance Through Reducing Thioredoxin-Interacting Protein (TXNIP) and Suppressing ER Stress in C2C12 Myotubes

**DOI:** 10.3389/fphar.2018.01180

**Published:** 2018-10-16

**Authors:** Mingxin Li, Yemin Zhang, Yingkang Cao, Deling Zhang, Le Liu, Yanghongyun Guo, Changhua Wang

**Affiliations:** Department of Pathology and Pathophysiology, Wuhan University School of Basic Medical Sciences, Wuhan, China

**Keywords:** icariin, insulin resistance, TXNIP, proteasome, skeletal muscle cells

## Abstract

Both thioredoxin-interacting protein (TXNIP) and endoplasmic reticulum (ER) stress are implicated in skeletal muscle insulin resistance. Icariin has been found to mimic insulin action in normal skeletal muscle C2C12 cells and display anti-diabetic properties in diet-induced obese mice. However, the underlying molecular mechanism remains to be well-established. Herein, we tested the hypothesis that the protective effects of icariin on free fatty acid-induced insulin resistance were attributed to its regulation on TXNIP protein levels and ER stress in skeletal muscle cells. We found that TXNIP mediated the saturated fatty acid palmitate (PA)-induced insulin resistance in C2C12 myotubes. Icariin treatment significantly restored PA-reduced proteasome activity resulting in reduction of TXNIP protein and suppression of ER stress, as well as improvement of insulin sensitivity. Proteasome inhibition by its specific inhibitor MG132 obviously abolished the inhibitory effect of icariin on PA-induced insulin resistance. In addition, MG132 supplementation markedly abrogated the impacts of icariin on ER stress and TXNIP-mediated downstream events such as inflammation and STAT3 phosphorylation. These results clearly indicate that icariin improves PA-induced skeletal muscle insulin resistance through a proteasome-dependent mechanism, by which icariin downregulats TXNIP levels and inhibits ER stress.

## Introduction

It has been demonstrated that the development and progression of diabetes and diabetic-related diseases are closely associated with insulin resistance, a pathophysiological condition characterized by an impaired insulin action in insulin-sensitizing tissues like liver, adipose tissue, and skeletal muscle. Skeletal muscle is responsible for up to 80% insulin-mediated glucose disposal under normal physiological condition (Thiebaud et al., 1982; DeFronzo et al., 1985). Thus, skeletal muscle insulin resistance plays a critical role in the development of type 2 diabetes. The elevated plasma free fatty acid (FFA) level is a well-known risk factor contributing to the initiation of skeletal muscle insulin resistance (Ye, 2007; Rachek, 2014). However, although an enormous amount of hypotheses has been postulated, more studies are still needed to elucidate the mechanisms underlying FFA-induced skeletal muscle insulin resistance.

The article "Icariin Ameliorates Palmitate-Induced Insulin Resistance Through Reducing Thioredoxin-Interacting Protein (TXNIP) and Suppressing ER Stress in C2C12 Myotubes" was retracted in 2023. Reasons: duplicated images; unreliable data; unreliable results or conclusions; concerns about the images.

Icariin (8-prenyl derivative of kaempferol 3,7-*O*-diglucoside) is a type of flavonoid extracted from the *Epimedium* genus (Liu et al., 2006). Despite no studies have been carried out on patients, icariin has usually been used for the treatment of erectile dysfunction in traditional Chinese medicine. Indeed, several *in vivo* animal studies have indicated that icariin may be a promising therapeutic agent for restoring erectile function (Liu et al., 2005, 2011; Wang et al., 2017). Currently, a growing number of *in vitro* and *in vivo* studies have also evidenced the multiple pharmacological activities of icariin. It could be used for the prevention or treatment of the various diseases such as neurodegenerative disorders, cardiovascular diseases, cancers, organ injuries, kidney diseases and etc., through multiple mechanisms including regulating inflammation, oxidative stress, apoptosis as well as angiogenesis (Schluesener and Schluesener, 2014; Li et al., 2015; Fang and Zhang, 2017).

Most interestingly, icariin exhibits anti-diabetic effects. It could reduce lipid accumulation in adipocytes (Han et al., 2016), inhibit adipocyte differentiation (Han et al., 2016), improve insulin sensitivity, glycemic control, and lipid metabolism in diet-induced obese (DIO) mice (Fu et al., 2015), and ameliorate diabetic complications such as diabetic retinopathy (Qi et al., 2011; Xin et al., 2012) and diabetic-related erectile dysfunction (Liu et al., 2011; Wang et al., 2017). In normal skeletal muscle C2C12 cells, icariin mimics insulin function. It could enhance adiponectin generation, activate AMPK, and sensitize insulin signaling, evidenced as an increase in IRS-1 phosphorylation and PI3K protein levels (Han et al., 2015). These findings suggest a novel mechanism by which icariin modulates insulin signaling. However, whether and how icariin affects FFA-induced skeletal muscle insulin resistance remains largely unknown.

In the present study, we investigated the impacts of icariin on palmitate (PA)-induced insulin resistance in C2C12 myotubes. We found that PA administration significantly increased the protein levels of thioredoxin-interacting protein (TXNIP), which has been suggested to negatively regulate insulin signaling. Icariin intervention improved PA-induced insulin resistance by promoting proteasome-dependent degradation of TXNIP and suppressing ER stress. This new finding should provide a better understanding of the molecular mechanism of icariin action.

The article "Icariin Ameliorates Palmitate-Induced Insulin Resistance Through Reducing Thioredoxin-Interacting Protein (TXNIP) and Suppressing ER Stress in C2C12 Myotubes" was retracted in 2023. Reasons: duplicated images; unreliable data; unreliable results or conclusions; concerns about the images.

## Materials and Methods

### Antibodies and Reagents

Antibodies against TXNIP (#14715), Akt (#2920), phosphor-Akt (Thr308) (#4056), AS160 (#2670), phosphor-AS160 (Ser588) (#8730), PDK1 (#13037), GLUT4 (#2213), PERK (#3192), IRE1α (#3294), CHOP (#5554), ATF6 (#65880), Histone H3 (#9715), IRS-1 (#2382), phosphor-IRS-1 (Ser307), JNK (#9252), phosphor-JNK (Thr183/Tyr185) (#4668), NF-κB p65 (#4764), phosphor-NF-κB p65 (Ser536) (#3033), and IκBα (#9242) were from Cell Signaling TECHNOLOGY (Beverly, MA, United States). Anti-PERK (phosphor T982) (ab192591), STAT3 (ab119352), STAT3 (phosphor Y705) (ab76315), and SOCS3 (ab16030) antibodies were obtained from Abcam, Inc. (Cambridge, MA, United States). Anti-IL-6 mouse monoclonal antibody (sc-57315) and normal mouse IgG (sc-2025) were purchased from Santa Cruz Biotechnology (Shanghai) Co., Ltd. (Shanghai, China). Insulin (91077C), palmitic acid (P5585), and icariin (I1286) were acquired from Sigma-Aldrich, Corp. (St. Louis, MO, United States). 2-Deoxy-D-2-[3H] glucose was obtained from HTA, Co. Ltd. (Beijing, China).

### Cells and Treatment

C2C12 myoblasts (CRL-1772^TM^) were obtained from American Type Culture Collection (ATCC, Manassas, VA, United States) and grown in DMEM (Cat #:30-2002, ATCC) containing 10% newborn calf serum (NCS) and 1% penicillin/streptomycin (P/S) in a humidified incubator with 5% CO_2_ and 95% air at 37°C.

C2C12 myotubes were produced by incubating C2C12 myoblasts in fresh DMEM with 0.1% NCS, 1% P/S, and 50 nmol/L insulin for 4 days (Conejo et al., 2001; Wang et al., 2009a).

Solution of palmitic acid was prepared as described previously (Wang et al., 2009a). C2C12 myotubes were starved serum for 4 h and then incubated with 0.5 mmol/L of PA for another 18 h to induce insulin resistance (Wang et al., 2009a). To assay insulin action, the cells were stimulated with 100 nmol/L insulin for a further 10 min.

### Small Interfering RNA (siRNA) and Transfection

The small interfering RNA (siRNA) was synthesized by QIAGEN China (Shanghai) Co. (Shanghai, China). C2C12 myotubes were transfected with 40 nmol/L siRNA for 72 h by using Lipofectamine RNAiMAX Transfection Reagent (Invitrogen, Carlsbad, CA, United States), according to the manufacturer’s protocol. The most effective sequences of siRNAs targeting mouse TXNIP (NM_001009935) and its paired control were as follows: 5′-GCAAACAGACTTTGGACTA-3′ and 5′-GCAACAGTCTTGGAAACTA-3′. Western blot was performed to measure the transfection efficiency.

### Preparation of Plasma Membrane and Nuclear Fractionation

The plasma membrane and nuclear fractionations were obtained by using Plasma Membrane Protein Extraction Kit (ab65400) (Abcam, Cambridge, MA, United States) and Nuclear/Cytosolic Fractionation Kit (AKR-171) (Cell Biolabs, Inc., San Diego, CA, United States), respectively. Western blot was performed to determine GLUT4 expression on plasma membrane and ATF6 protein levels in nuclear homogenates. The membrane marker cadherin and nuclear histone H3 served as controls, respectively.

The article "Icariin Ameliorates Palmitate-Induced Insulin Resistance Through Reducing Thioredoxin-Interacting Protein (TXNIP) and Suppressing ER Stress in C2C12 Myotubes" was retracted in 2023. Reasons: duplicated images; unreliable data; unreliable results or conclusions; concerns about the images.

### Glucose Uptake Determination

Glucose uptake was measured by 2-deoxy-D-2-[3H] glucose as described previously (Wang et al., 2009b; Zhang et al., 2015).

### Quantitative RT-PCR

Total RNA was isolated from C2C12 myotubes using TRIzol reagent (Invitrogen, Carlsbad, CA, United States) and complementary DNAs were synthesized by Superscript II Reverse Transcriptase (Invitrogen) according to the manufacturer’s protocol. Quantitative real-time RT-PCR was performed using QuantiTect SYBR Green PCR Kit (Cat No. 204143, QIAGEN, Shanghai) and an Applied Biosystems 7500 Real-Time PCR system (Applied Biosystems, Foster City, CA, United States). The oligonucleotide primer sequences used in this study include mouse IL-6 (NM_031168): forward 5′-GGTGACAACCACGGCCTTCCC-3′, reverse 5′-AAGCCTCCGACTTGTGAAGTGGT-3′; mouse TXNIP (NM_001009935): forward 5′-CATGAGGCCTGGAAACAAAT-3′, reverse 5′-ACTGGTGCCATTAGGTCAGG-3′; mouse CHOP (NM_007837.4): forward 5′-CTGCCTTTCACCTTGGAGAC-3′, reverse 5′-CGTTTCCTGGGGATGAGATA-3′; mouse GAPDH (NM_008084): forward 5′-TGGAAAGCTGTGGCGTGAT-3′, reverse 5′-TGCTTCACCACCTTCTTGAT-3′. The 2^-ΔΔC^t method was used for relative quantification of gene expression and GAPDH was used as an internal control for normalization. All samples were analyzed in triplicate.

### Proteasomal Peptidase Activity Assays

The chymotrypsin-like activity of 20S proteasome was determined using synthetic fluorogenic peptide substrate Suc-LLVY-AMC (Boston Biochem, Cambridge, MA, United States) as described previously (Zhang et al., 2015; Ye et al., 2017). The fluorescence intensity was recorded at an excitation wavelength of 350 nm and emission wavelength of 440 nm using fluorescence spectrometer (Perkin Elmer precisely LS 55, Billerica, MA, United States).

### Western Blot

The abundances of proteins or phosphorylated proteins were detected by western blot as described previously (Wang et al., 2009a; Zhang et al., 2015; Ye et al., 2017).

### Statistical Analysis

The data shown represent the means ± standard deviation (SD). The differences between the groups were examined for statistical significance using analysis of variance (ANOVA), followed by a Newman–Keuls *post hoc* test. A *p*-value < 0.05 is regarded as statistically significant. The figures are the representative of at least four independent experiments with similar results.

The article "Icariin Ameliorates Palmitate-Induced Insulin Resistance Through Reducing Thioredoxin-Interacting Protein (TXNIP) and Suppressing ER Stress in C2C12 Myotubes" was retracted in 2023. Reasons: duplicated images; unreliable data; unreliable results or conclusions; concerns about the images.

## Results

### Icariin Mitigated PA-Induced Insulin Resistance

To observe the potential impacts of icariin on insulin resistance, C2C12 myotubes were starved serum for 4 h and then treated with or without 0.5 mmol/L of PA in the presence or absence of 25, 50, or 100 μmol/L icariin for 18 h, followed by stimulation with or without 100 nmol/L insulin for 10 min. As shown in **Figure 1**, icariin treatment protected C2C12 myotubes against PA-induced insulin resistance in a dose-dependent manner, as demonstrated by the gradual recoveries of insulin-stimulated phosphorylation of Akt at Thr308 and of its downstream substrate AS160 (**Figures 1A,B**). Consistence with this result, the cells treated with a combination of 0.5 mmol/L PA and 50 μmol/L icariin displayed the increased GLUT4 expressions on plasma membrane (**Figures 1C,D**) and the enhanced 2-DG uptake (**Figure 1E**) under stimulation with insulin, when compared with PA treatment alone. These results clearly indicated that icariin attenuated the deleterious effects of PA on insulin signaling in C2C12 myotubes.

**FIGURE 1:** Impacts of icariin on PA-induced insulin resistance in C2C12 myotubes. **(A,B)** Dose–response effect of icariin (ICA) on insulin (INS)-stimulated phosphorylation of Akt T308 and AS160. **(C,D)** Effect of ICA on INS-stimulated GLUT4 translocation on plasma membrane. **(E)** Effect of ICA on INS-stimulated 2-deoxy-D-glucose (2-DG) uptake. *N* = 4. ^∗∗^*p* < 0.01, ^∗∗∗^*p* < 0.001 vs. control (Cont)/INS group; ##*p* < 0.01, ###*p* < 0.001 vs. PA/INS group.

### TXNIP Mediated the Inhibitory Effects of PA on Insulin Signaling

When serum-starved C2C12 myotubes were treated with 0.5 mmol/L of PA for 18 h, we found that PA exposure significantly increased the abundance of TXNIP protein (**Figure 2A**). To elucidate the association between TXNIP and PA-induced insulin resistance, TXNIP in C2C12 myotubes was silenced by siRNA techniques. Knockdown or control C2C12 myotubes were starved serum for 4 h and then treated with 0.5 mmol/L PA for another 18 h, followed by stimulated with or without 100 nmol/L insulin for 10 min. We found that TXNIP knockdown markedly increased insulin-stimulated Akt phosphorylation at Thr308 (**Figures 2B,C**), GLUT4 translocation on plasma membrane (**Figure 2D**), and 2-DG uptake (**Figure 2E**), which is consistent with the previous study showing that TXNIP plays critical role in PA-induced insulin resistance (Mandala et al., 2016).

**FIGURE 2:** Impacts of TXNIP on PA-induced insulin resistance in C2C12 myotubes. **(A)** Effect of PA on TXNIP protein levels. **(B,C)** Effect of TXNIP knockdown on insulin (INS)-stimulated Akt phosphorylation. **(D)** Effect of TXNIP knockdown on INS-stimulated GLUT4 translocation on plasma membrane. **(E)** Effect of TXNIP knockdown on INS-stimulated 2-deoxy-D-glucose (2-DG) uptake. *N* = 4. ^∗∗^*p* < 0.01 vs. control (Cont) group or the indicated group.

The article "Icariin Ameliorates Palmitate-Induced Insulin Resistance Through Reducing Thioredoxin-Interacting Protein (TXNIP) and Suppressing ER Stress in C2C12 Myotubes" was retracted in 2023. Reasons: duplicated images; unreliable data; unreliable results or conclusions; concerns about the images.

### Icariin Accelerated TXNIP Degradation Through the Proteasome System

To investigate whether icariin affects PA-induced TXNIP expression, serum-starved C2C12 myotubes were incubated with 0.5 mmol/L of PA in the presence or absence of 50 μmol/L icariin for 18 h. Western blot and qRT-PCR were performed to detect the levels of TXNIP protein or mRNA, respectively. As shown in **Figures 3A,B**, icariin treatment significantly reduced TXNIP protein levels whereas TXNIP mRNA levels remained unchanged when compared with PA treatment alone. Then, we tested the impact of translation inhibitor cycloheximide (CHX) on the stability of TXNIP protein. Serum-starved C2C12 myotubes were treated with or without 50 μmol/L icariin for 18 h, and then incubated with 100 μmol/L of CHX for 15 or 30 min. We found that the combined treatment of CHX and icariin accelerated TXNIP reduction comparing with CHX treatment alone (**Figures 3C,D**), suggesting that icariin suppressed TXNIP expression through a post-translation mechanism.

**FIGURE 3:** Impacts of icariin on TXNIP expression in PA-treated C2C12 myotubes. **(A)** Effect of icariin (ICA) on TXNIP protein levels. **(B)** Effect of ICA on TXNIP mRNA levels. **(C,D)** Effect of ICA on the stability of TXNIP protein (chase experiments). **(E,F)** Effect of the inhibitors of proteasome and autophagy on TXNIP protein levels. **(G)** Effect of ICA on the chymotrypsin-like (ChL) activity of proteasome. *N* = 4. ^∗∗^*p* < 0.01, ^∗∗∗^*p* < 0.001 vs. control (Cont) or the indicated group; ##*p* < 0.01 vs. PA group; §*p* > 0.05 vs. the indicated group.

The ubiquitin–proteasome system (UPS) and autophagy are responsible for the degradation of most intracellular proteins (Wong and Cuervo, 2010; Varshavsky, 2017). To address the mechanism underlying TXNIP down-regulation by icariin treatment, serum-starved C2C12 myotubes were pre-treated with 5 μmol/L MG132 (a specific UPS inhibitor) or 100 nmol/L bafilomycin A1 (BFA, a selective autophagy inhibitor) for 1 h, and then incubated with 0.5 mmol/L PA in the presence or absence of 50 μmol/L icariin for another 18 h. We found that icariin-reduced TXNIP expression was restored by MG132 treatment but not by BFA administration (**Figures 3E,F**). In addition, icariin treatment significantly enhanced the chymotrypsin-like activity of proteasome when compared with PA treatment alone (**Figure 3G**).

Taken together, these results indicate that icariin activated proteasome activities leading to TXNIP degradation.

The article "Icariin Ameliorates Palmitate-Induced Insulin Resistance Through Reducing Thioredoxin-Interacting Protein (TXNIP) and Suppressing ER Stress in C2C12 Myotubes" was retracted in 2023. Reasons: duplicated images; unreliable data; unreliable results or conclusions; concerns about the images.

### Icariin Reduced PA-Induced ER Stress

TXNIP levels could also be regulated by ER stress (Lerner et al., 2012; Oslowski et al., 2012). To test this possibility, C2C12 myotubes were starved serum for 4 h and then treated with 0.5 mmol/L of PA in the presence or absence of 50 μmol/L icariin for another 18 h. We found that the PA-increased expressions of protein markers of ER stress like phosphorylated PERK, phosphorylated IRE1, and CHOP were greatly inhibited by icariin treatment (**Figures 4A,B**). Consistently, PA-increased levels of ATF6 protein in nuclear and CHOP mRNA were significantly mitigated by icariin administration (**Figures 4C,D**). Icariin treatment also markedly inhibited phosphorylation of JNK and IRS-1 at Ser307 (**Figures 4E,F**), which has been suggested to mediate ER stress-induced insulin resistance (Ozcan et al., 2004; Nakatani et al., 2005).

**FIGURE 4:** Impacts of icariin on ER stress in PA-treated C2C12 myotubes. **(A,B)** Effect of icariin (ICA) on the protein levels of ER stress markers. **(C)** Effect of ICA on CHOP mRNA levels. **(D)** Effect of ICA on the protein levels of ATF6 in nuclear. **(E,F)** Effect of ICA on phosphorylation of JNK and IRS-1. *N* = 4. ^∗∗^*p* < 0.01, ^∗∗∗^*p* < 0.001 vs. control (Cont) group; ^#^*p* < 0.05, ^##^*p* < 0.01, ^###^*p* < 0.001 vs. PA group.

### Icariin Suppressed PA-Induced Inflammation and STAT3 Phosphorylation

When serum-starved C2C12 myotubes were incubated with 0.5 mmol/L of PA in the presence or absence of 50 μmol/L icariin for 18 h, we found that icariin-treated cells showed the decreased phosphorylation of NF-κB p65 and the increased expression of IκB protein when compared with PA treatment alone (**Figures 5A,B**). In addition, PA-increased IL-6 mRNA expressions were also obviously suppressed by icariin administration (**Figure 5C**).

**FIGURE 5:** Impacts of icariin on inflammation in PA-treated C2C12 myotubes. **(A,B)** Effect of icariin (ICA) on NF-κB p65 phosphorylation and IκB protein levels. **(C)** Effect of ICA on IL-6 mRNA levels. *N* = 4. ^∗∗^*p* < 0.01, ^∗∗∗^*p* < 0.001 vs. control (Cont) group; ##*p* < 0.01 vs. PA group.

Constitutive STAT3 activation has been implicated in skeletal muscle insulin resistance in type 2 diabetes (Mashili et al., 2013). We hence used the same experiments as described above to study whether STAT3 is involved in PA-induced insulin resistance and how icariin affects it. As shown in **Figure 6**, PA-increased STAT3 phosphorylation was greatly suppressed by icariin administration (**Figures 6A,B**). Considering that IL-6 is a major activator of STAT3 (Jiang et al., 2013; Harder-Lauridsen et al., 2014), we wondered whether IL-6 mediates icariin action on insulin signaling. Serum-starved C2C12 myotubes were treated with 0.5 mmol/L PA in the presence or absence of 50 μmol/L icariin or 5 μg/ml IL-6-neutralizing antibodies for 18 h. The same concentration of normal IgG served as controls. We found that PA-enhanced STAT3 phosphorylation and SOCS3 protein levels remained unchanged under treatment with IL-6 antibody (**Figures 6C,D**), suggesting that icariin-suppressed STAT3 phosphorylation was independent on IL-6.

The article "Icariin Ameliorates Palmitate-Induced Insulin Resistance Through Reducing Thioredoxin-Interacting Protein (TXNIP) and Suppressing ER Stress in C2C12 Myotubes" was retracted in 2023. Reasons: duplicated images; unreliable data; unreliable results or conclusions; concerns about the images.

**FIGURE 6:** Impacts of icariin on STAT3 signaling in PA-treated C2C12 myotubes. **(A,B)** Effect of icariin (ICA) on STAT3 phosphorylation and SOCS3 protein levels. **(C,D)** Effect of IL-6-neutralizing antibody (IL-6 Ab) on STAT3 phosphorylation and SOCS3 protein levels. **(E,F)** Effect of TXNIP knockdown on STAT3 phosphorylation and SOCS3 protein levels. *N* = 4. ^∗∗∗^*p* < 0.001 vs. control (Cont) or scramble control (SC) group; ^##^*p* < 0.01, ^###^*p* < 0.001, vs. PA or SC/PA group; §*p* > 0.05 vs. PA group.

To figure out the role of TXNIP in PA-enhanced STAT3 phosphorylation, TXNIP-knockdown C2C12 myotubes were starved serum for 4 h and then treated with 0.5 mmol/L of PA in the presence or absence of 50 μmol/L icariin for another 18 h. As shown in **Figures 6E,F**, PA-induced STAT3 phosphorylation was significantly inhibited by TXNIP silence, suggesting TXNIP mediated PA-stimulated STAT3 phosphorylation.

### Proteasome Inhibition Abolished Icariin Action on PA-Induced Insulin Resistance

To further characterize the relationship between icariin-activated proteasome activity and insulin resistance, we tested the effects of proteasome inhibition on ER stress, inflammation, and STAT3 phosphorylation. Serum-starved C2C12 myotubes were pretreated with or without 5 μmol/L MG132 for 1 h and then incubated with 0.5 mmol/L of PA in the presence or absence of 50 μmol/L icariin for another 18 h. As shown in **Figure 7**, MG132 administration obviously recovered the expression levels of ER stress markers (**Figures 7A,B**), phosphorylated p65 and IκB protein (**Figures 7C,D**), and phosphorylated STAT3 (**Figures 7E,F**), when compared with a combination treatment of PA and icariin.

**FIGURE 7:** Impacts of proteasome inhibition on ER stress, inflammation, and STAT3 phosphorylation in C2C12 myotubes cotreated with PA and icariin (ICA). **(A,B)** Effect of MG132 on the protein levels of ER stress markers. **(C,D)** Effect of MG132 on p65 phosphorylation and IκB protein levels. **(E,F)** Effect of MG132 on STAT3 phosphorylation and SOCS3 protein levels. *N* = 4. ^∗∗^*p* < 0.01 vs. the indicated group; §*p* > 0.05 vs. the indicated group.

The article "Icariin Ameliorates Palmitate-Induced Insulin Resistance Through Reducing Thioredoxin-Interacting Protein (TXNIP) and Suppressing ER Stress in C2C12 Myotubes" was retracted in 2023. Reasons: duplicated images; unreliable data; unreliable results or conclusions; concerns about the images.

Under stimulation with 100 nmol/L insulin for 10 min, MG132 treatment also markedly mitigated the effects of icariin on insulin-stimulated Akt phosphorylation at Thr308 (**Figures 8A,B**), GLUT4 translocation on plasma membrane (**Figures 8C,D**), and 2-DG uptake (**Figure 8E**).

**FIGURE 8:** Impacts of proteasome inhibition on insulin signaling in C2C12 myotubes cotreated with PA and icariin (ICA). **(A,B)** Effect of MG132 on insulin (INS)-stimulated Akt phosphorylation. **(C,D)** Effect of MG132 on INS-stimulated GLUT4 translocation on plasma membrane. **(E)** Effects of MG132 on INS-stimulated 2-deoxy-D-glucose (2-DG) uptake. *N* = 4. ^∗∗^*p* < 0.01, ^∗∗∗^*p* < 0.001 vs. the indicated group; §*p* > 0.05 vs. the indicated group.

These results suggest that proteasome inhibition abrogated the protective effects of icariin on PA-induced ER stress, inflammation, STAT3 phosphorylation as well as insulin resistance.

## Discussion

The insulin-sensitizing action of icariin has been shown in normal skeletal muscle C2C12 cells and DIO mice (Fu et al., 2015; Han et al., 2015). However, the underlying mechanism remains to be fully elucidated. In the present study, we found that TXNIP mediated PA-induced insulin resistance in C2C12 myotubes (**Figure 2**). Icariin administration brought about a reduction in TXNIP protein via a proteasome dependent mechanism (**Figure 3**) and a significant improvement in ER stress (**Figure 4**) and insulin sensitivity (**Figure 1**). Proteasome inhibition by its specific inhibitor MG132 abolished the beneficial effects of icariin on insulin signaling in the PA-treated C2C12 myotubes (**Figure 8**). MG132 supplementation also abrogated icariin’s impacts on ER stress and TXNIP-mediated downstream events such as inflammation and STAT3 phosphorylation (**Figure 7**). Our results suggest that icariin protected skeletal muscle cells against PA-induced insulin resistance by inducing proteasome-dependent degradation of TXNIP and suppressing ER stress.

Previous studies have reported that high levels of TXNIP are responsible for pancreatic β cell apoptosis and peripheral insulin resistance (Alhawiti et al., 2017; Kawamoto et al., 2018). In skeletal muscle cells, TXNIP mediated PA-induced insulin resistance (Mandala et al., 2016). On the contrary, total and muscle-specific TXNIP knockdown mice exhibit increased insulin sensitivity and are protected against diet-induced insulin resistance and diabetes (Hui et al., 2008; Chutkow et al., 2010; Alhawiti et al., 2017). In addition, caloric restriction-induced improvement of insulin sensitivity is achieved by lowering insulin-stimulated TXNIP levels, independently on mitochondrial oxidative capacity and metabolite levels like ceramide, diacylglycerol, or amino acid in skeletal muscle (Johnson et al., 2016). These findings strongly demonstrated that TXNIP negatively regulates insulin signaling. Consistently, our results confirmed that PA stimulated TXNIP expression (**Figure 2A**) (Mandala et al., 2016). Genetic or pharmacological inhibition of TXNIP by siRNA or icariin significantly mitigated PA-induced insulin resistance (**Figures 1–3**), further backing up previous speculation that TXNIP in skeletal muscle is a promising therapeutic target for prevention and treatment of insulin resistance and diabetes.

The article "Icariin Ameliorates Palmitate-Induced Insulin Resistance Through Reducing Thioredoxin-Interacting Protein (TXNIP) and Suppressing ER Stress in C2C12 Myotubes" was retracted in 2023. Reasons: duplicated images; unreliable data; unreliable results or conclusions; concerns about the images.

It has been documented that TXNIP are regulated by ER stress and proteasome activity. TXNIP mRNA levels can be augmented by ER stress through the PERK and IRE1 pathways (Anthony and Wek, 2012). On the other hand, TXNIP undergoes proteasomal degradation in various types of cells (Shao et al., 2010; Zhang et al., 2010). In the present study, we found that icariin treatment significantly restored PA-reduced proteasome activity (**Figure 3G**) and suppressed PA-enhanced ER stress (**Figures 4A,B**). However, the mRNA levels of TXNIP remained unchanged in the cells treated with PA alone or a combination of PA and icariin (**Figure 3B**). Combined with our findings showing that inhibition of ER stress by 4-PBA did not changes PA-induced protein expressions of TXNIP (Data not shown), our results indicate that the reduction of TXNIP protein is mainly attributed to icariin-improved proteasome activity.

Icariin possesses the properties of phosphodiesterase type 5 (PDE5) inhibitors and inhibits all three PDE5 isoforms (Xin et al., 2003; Rahimi et al., 2010). It is becoming clear that PDE5 inhibition will accumulate the intracellular cGMP concentration leading to the activation of protein kinase G (PKG) (Das et al., 2008), which has been found to stimulate proteasome activities through a mechanism for post-translational modifications of proteasome subunits (Ranek et al., 2013). Indeed, icariin has been evidenced to increase the expression levels of some proteasome subunits like proteasome subunit-alpha type 6 and type 2, and reverse the inhibitory impacts of proteasome inhibitor epoxomicin on proteasome activity (Zhu et al., 2011). In addition, PDE5 is expressed in skeletal muscle and in proliferating and differentiated C2C12 cells (Loughney et al., 1998; Sabatini et al., 2011). PDE5 activity is also closely associated with glucose metabolism in C2C12 cells (Sabatini et al., 2011). Thus, there is a possibility that PDE5/cGMP/PKG signaling mediates icariin action on proteasome activity. More studies are required to further confirm this hypothesis.

The article "Icariin Ameliorates Palmitate-Induced Insulin Resistance Through Reducing Thioredoxin-Interacting Protein (TXNIP) and Suppressing ER Stress in C2C12 Myotubes" was retracted in 2023. Reasons: duplicated images; unreliable data; unreliable results or conclusions; concerns about the images.

Recent studies have suggested that both inflammation and constitutive STAT3 phosphorylation contribute significantly to PA-induced skeletal muscle insulin resistance (Coll et al., 2008, 2010; Mashili et al., 2013). In the present study, we found that PA-induced inflammation and STAT3 hyperphosphorylation were significantly inhibited by icariin intervention (**Figures 5, 6**), whereas these inhibitory effects were almost completely abolished by MG132 treatment (**Figure 7**). Given that icariin-reduced TXNIP levels were greatly restored by MG132 treatment (**Figures 3E,F**) and that TXNIP knockdown mitigated PA-stimulated STAT3 phosphorylation (**Figures 6E,F**), it is reasonable to postulate that the proteasome-dependent degradation of TXNIP is responsible for the inhibitory impacts of icariin on inflammation and excessive STAT3 phosphorylation.

The causal relationship between TXNIP and inflammation has been well-elucidated in various diseases including type 2 diabetes (Lerner et al., 2012; Oslowski et al., 2012; Shah et al., 2013; Chong et al., 2014). A question that remains to be addressed is how TXNIP regulates STAT3 phosphorylation. It has been suggested that IL-6/STAT3 signaling is closely associated with insulin sensitivity (Jiang et al., 2013; Harder-Lauridsen et al., 2014). Previous study has reported that PA exposure markedly enhances mRNA levels and secretion of IL-6 in C2C12 myotubes, suggesting that IL-6 mediates inhibitory effects of palmitate on insulin signaling (Jové et al., 2005). Consistent with this finding, we found that icariin treatment significantly suppressed PA-induced IL-6 mRNA (**Figure 5C**). However, PA-induced STAT3 phosphorylation was significantly inhibited by icariin treatment but not by IL-6 antibodies (**Figures 6C,D**). Our results suggest that PA-activated STAT3 phosphorylation is independent on IL-6 stimulation, which is consistent with previous study showing that chronic IL-6 stimulation does not affect STAT3 phosphorylation in skeletal muscle cells (Mashili et al., 2013). It is noteworthy that TXNIP upregualtion has been found to impair activity of STAT3 in INS-1 cells and cardiac myocytes (Xu et al., 2013; Hu et al., 2015). Conversely, previous study also evidences that TXNIP reduces miR-124a levels (Jing et al., 2014), a microRNA directly binding to the 3′-UTR region of STAT3 leading to the reduction of STAT3 protein and mRNA (Lu et al., 2013; Nagata et al., 2014). Therefore, TXNIP may stimulate STAT3 signaling through enhancing STAT3 levels. In the present study, neither PA nor icariin affects STAT3 protein levels (**Figure 6A**). However, PA-stimulated STAT3 phosphorylation was significantly inhibited by TXNIP siRNA and icariin supplementation (**Figure 6**). In addition, proteasome inhibition by MG132 markedly diminished the impacts of icariin on STAT3 phosphorylation (**Figures 7E,F**). Given that icariin treatment induced a proteasome-dependent reduction of TXNIP protein, these data suggest that PA-stimulated STAT3 phosphorylation is mediated by TXNIP. However, more studies are required to investigate the underlying mechanism.

The article "Icariin Ameliorates Palmitate-Induced Insulin Resistance Through Reducing Thioredoxin-Interacting Protein (TXNIP) and Suppressing ER Stress in C2C12 Myotubes" was retracted in 2023. Reasons: duplicated images; unreliable data; unreliable results or conclusions; concerns about the images.

Despite proteasome-dependent degradation of important molecules in the insulin signaling pathway has been found to contribute to insulin resistance (Wing, 2008), a growing number of studies have evidenced that normal proteasome function is necessary for maintaining insulin sensitivity. For example, reduced proteasome activity and insulin resistance coexist in the liver of obese and diabetic mice, adipose tissues of DIO mice, and PA-treated 3T3-L1 adipocytes (Otoda et al., 2013; Díaz-Ruiz et al., 2015). Silence of proteasome activator 28 (PA28) causes the glucose intolerance and hepatic insulin resistance (Otoda et al., 2013). Furthermore, pharmacological inhibition of proteasome has been found to impair insulin signaling in adipocytes and hepatocytes (Otoda et al., 2013; Díaz-Ruiz et al., 2015), or further exacerbates insulin resistance in myotubes from type 2 diabetic patients (Al-Khalili et al., 2014). Perhaps the most reasonable explanation for these findings is that proteasome deficiency will accumulate the ubiquitinated proteins in ER lumen resulting in ER stress and unfold protein response (UPR) (Cybulsky, 2013; Otoda et al., 2013), which leads to activation of JNK/IRS-1 pathway and subsequent insulin resistance (Ozcan et al., 2004; Nakatani et al., 2005). Thus, maintenance of proteasome activity by icariin should attenuate PA-induced insulin resistance in C2C12 myotubes partly through suppressing ER stress (**Figure 4**).

Taken together, our results revealed that icariin heightened proteasome-dependent degradation of TXNIP and inhibited ER stress, leading to improvement of PA-induced insulin resistance in skeletal muscle cells (**Figure 9**). This new finding provides a novel mechanism by which icariin produces its anti-diabetic effects.

**FIGURE 9:** Schematic diagram of icariin regulation upon PA-induced insulin resistance. Proteasome functions as a key role in PA-induced insulin resistance in C2C12 myotubes. Dysfunction of proteasome facilitates ER stress and promotes an increase of TXNIP protein levels. Excessive TXNIP contributes to inflammatory response and hyperactivation of STAT3 leading to insulin resistance. In addition, ER stress induces insulin resistance through inflammation and JNK/IRS-1 pathway. The precise mechanism that regulates proteasome remains unclear; however, the improvement of proteasome activity by icariin administration results in degradation of TXNIP protein and attenuation of ER stress, both of which contribute to improvement of insulin resistance.

The article "Icariin Ameliorates Palmitate-Induced Insulin Resistance Through Reducing Thioredoxin-Interacting Protein (TXNIP) and Suppressing ER Stress in C2C12 Myotubes" was retracted in 2023. Reasons: duplicated images; unreliable data; unreliable results or conclusions; concerns about the images.

### Limitations

In the present study, we clearly elucidate the molecular mechanism by which icariin protects C2C12 myotubes against PA-induced insulin resistance. However, although some methods such as proteasomal peptidase activity assay, glucose uptake measure, and qRT-PCR were used in the experiments, the majority of the results were based on western blotting analysis. It would be better to provide more evidences to make results further solid. For example, immunofluorescence technique could be used to detect or localize a specific protein in cytosol or on plasma membrane.

In addition, the concentration of icariin used in this study is relative high. Previous studies have evidenced that the cytotoxicity of icariin is associated with cell types, the physiological or pathophysiological status of cells, concentration or duration of icariin administration, and others. For instance, icariin significantly induces cell apoptosis and inhibits cell proliferation in various types of cancer cells (Tan et al., 2016). In human bone mesenchymal stem cells, cell survivals are promoted by low concentration but mitigated by high concentration of icariin (Wang et al., 2018). Interestingly, icariin at concentration of 150 or 200 μmol/L protects adipose derived mesenchymal stem cells against H_2_O_2_-induced cellular damages (Wang et al., 2017). Using MTT assay method, a cellular viability assay commonly used to monitor drug toxicity, we also found that icariin has no obvious toxicity to C2C12 myotubes (**Supplementary Figure S1**), which is partly consistent with previous study showing that icariin at the concentration of 50 or 100 μmol/L significantly increases cell viabilities in insulin-sensitizing 3T3-L1 cells (Han et al., 2016). Thence, icariin shows low toxicity or no obvious adverse effects to normal cells (Tan et al., 2016). However, the high dose may limit its application in clinical practice. Further studies are necessary to gain more potent derivatives from icariin.

## Author Contributions

CW and ML designed the studies. ML, YZ, YC, DZ, LL, and YG performed the experiments. CW, ML, and YZ conducted statistical analyses. CW wrote the manuscript. All authors approved submission of the manuscript.

## Conflict of Interest Statement

The authors declare that the research was conducted in the absence of any commercial or financial relationships that could be construed as a potential conflict of interest.
